# Neurexin-2 restricts synapse numbers and restrains the presynaptic release probability by an alternative splicing-dependent mechanism

This article has been retracted.

**DOI:** 10.1073/pnas.2300363120

**Published:** 2023-03-24

**Authors:** Pei-Yi Lin, Lulu Y. Chen, Peng Zhou, Sung-Jin Lee, Justin H. Trotter, Thomas C. Südhof

**Affiliations:** ^a^Department of Molecular and Cellular Physiology, Stanford University School of Medicine, Stanford, CA 94305; ^b^HHMI, Stanford University School of Medicine, Stanford, CA 94305

**Keywords:** neurexin, synapse formation, alternative splicing, neurotransmitter release, synaptic transmisssion

## Abstract

α- and β-neurexins are extensively alternatively spliced, presynaptic cell-adhesion molecules that are thought to organize synapse assembly. However, recent data revealed that, in the hippocampus in vivo, the deletion of one neurexin isoform, *Nrxn2*, surprisingly increased excitatory synapse numbers and enhanced their presynaptic release probability, suggesting that *Nrxn2* restricts, instead of enabling, synapse assembly. To delineate the synaptic function and mechanism of action of *Nrxn2*, we examined cultured hippocampal neurons as a reduced system. In heterologous synapse formation assays, different alternatively spliced Nrxn2β isoforms robustly promoted synapse assembly similar to Nrxn1β and Nrxn3β, consistent with a general synaptogenic function of neurexins. Deletion of *Nrxn2* from cultured hippocampal neurons, however, caused a significant increase in synapse density and release probability, replicating the in vivo data that suggested a synapse-restricting function. Rescue experiments revealed that two of the four Nrxn2β splice variants (Nrxn2β-SS4+/SS5− and Nrxn2β-SS4+/SS5+) reversed the increase in synapse density in *Nrxn2*-deficient neurons, whereas only one of the four Nrxn2β splice variants (Nrxn2β-SS4+/SS5+) normalized the increase in release probability in *Nrxn2*-deficient neurons. Thus, a subset of *Nrxn2* splice variants restricts synapse numbers and restrains their release probability in cultured neurons.

## Significance

Previous in vivo studies showed that neurexin-2 unexpectedly regulates synaptic connectivity in hippocampal circuits not by inducing, but by repressing excitatory synapses. The present study demonstrates that as assessed by heterologous synapse formation experiments, a commonly used in vitro synaptogenesis assay, neurexin-2 powerfully induces synapse formation. However, neurexin-2 deletions nevertheless increased the number and the release probability of synapses in cultured hippocampal neurons, indicating a synapse-restricting function consistent with the in vivo results. Rescue experiments revealed that the two phenotypes of the neurexin-2 deletion were differentially reversed by distinct combinations of neurexin-2βsplice variants, suggesting a dual restrictive mechanism of neurexin-2 in synaptic connectivity that differs from that of other neurexins and that is regulated by alternative splicing of neurexin-2.

Synapses connect neurons into circuits that process information. Synapses not only transfer a signal from one neuron to the next, but also process that signal computationally during transfer. Synapses exhibit diverse computational properties that are specified by the identities of the pre- and postsynaptic neurons, with likely hundreds of types of synapses formed in brain. Moreover, synapses are dynamic. In contrast to the neurons that make them, synapses are continuously restructured and remade throughout life, and are further tuned by synaptic plasticity and neuromodulators. In recent years, a detailed understanding of the basic properties and the machinery of synaptic transmission has been achieved, but the processes that govern synapse assembly, synapse elimination/replacement, and synaptic plasticity remain enigmatic.

Cell biologically, synapses are intercellular junctions specialized for information processing. As intercellular junctions, synapses are controlled by adhesion molecules (1, 2). Among these, presynaptic neurexins are likely the most important regulators of synapse properties (reviewed in refs. 3 and 4). Neurexins are encoded in vertebrates by three genes (*Nrxn1*-*Nrxn3* in mice), each of which has independent promoters for longer α-neurexins and shorter β-neurexins (5–8). In addition, a third promoter drives transcription of an additional even shorter *Nrxn1* isoform, Nrxn1γ, whereas the *Nrxn2* or *Nrxn3* genes lack this third promoter (9). Neurexins are highly homologous to each other in their primary sequences, and all neurexins are subject to extensive alternative splicing generating thousands of isoforms (10–12). Specifically, α-neurexins contain 6 canonical sites of alternative splicing (SS1-SS6), of which only SS6 is missing in Nrxn2α, while β-neurexins contain only 2 canonical sites of alternative splicing (SS4 and SS5).

Unexpectedly in view of their high degree of sequence homology, recent studies revealed that in subiculum synapses of the hippocampal formation, *Nrxn1* alternative splicing at SS4 regulates N-methyl-D-aspartate receptor (NMDAR)-type glutamate receptors (NMDARs), *Nrxn2* alternative splicing at SS4 has no effect on either NMDARs or α-amino-3-hydroxy-5-methyl-4-isoxazolepropionic acid receptor (AMPA)-type glutamate receptors (AMPARs), and *Nrxn3* alternative splicing at SS4 controls AMPARs (13–16). These observations demonstrated that alternative splicing of Nrxn1 and Nrxn3 at SS4 is physiologically important and indicated that the three neurexin isoforms can perform distinct roles at the same synapse. However, they also raised the question of what SS4-regulated function Nrxn2 might perform. Indeed, despite a large number of publications investigating neurexins (>1,400 papers as of 2022), only a few studies examined *Nrxn2*. *Nrxn2* is more distant evolutionarily from *Nrxn1* and *Nrxn3* than these two genes are to each other and its gene is smaller than that of *Nrxn1* and *Nrxn3* (5). We recently observed that in vivo deletions of *Nrxn2* induced a dramatic increase in synapse numbers and release probability in excitatory CA1-region synapses of the hippocampus (17), which was unexpected in view of the generally accepted notion that neurexins promote synapse assembly (3, 4). This finding suggested that *Nrxn2* acts to restrain synaptic connectivity but differed from those of an earlier study on another strain of *Nrxn2*-mutant mice which found that mutation of the *Nrxn2* gene decreases the miniature excitatory postsynaptic currents (mEPSC) frequency and the paired-pulse ratio of evoked responses of cortical synapses without changing synapse numbers (18). However, it is unclear whether the *Nrxn2*-mutant mice used in the earlier study (18) exhibit a decrease in *Nrxn2* expression since these *Nrxn2*-mutant mice were generated in our laboratory but could not be validated because of an apparent chromosomal rearrangement.

Our finding that the *Nrxn2* deletion increases synaptic connectivity was entirely dependent on in vivo manipulations that might have produced indirect effects (17). Given this fact and in view of the differences between the reported phenotypes of the *Nrxn2* deletion vs. the *Nrxn2* mutation (18), we here set out to leverage a less complex system, cultured neurons, to test whether *Nrxn2* exerts a pro- or anti-synaptogenic function. Moreover, since the *Nrxn2* deletion in vivo increased both synapse numbers and the release probability in the hippocampus (17) and since neurexins are generally regulated by alternative splicing, we asked whether the two *Nrxn2* effects on synapse numbers and release probability might be mediated by different splice variants of *Nrxn2*. Our results demonstrate that the conditional deletion of *Nrxn2* in cultured neurons causes a large increase in both synapse density and presynaptic release probability, confirming the in vivo results, and that these phenotypes are differentially rescued by *Nrxn2* splice variants, indicating that the two repressive functions of *Nrxn2* are mediated by distinct molecular mechanisms.

## Results

### *Nrxn2* Is Synaptogenic in Heterologous Synapse Formation Assays.

Heterologous synapse formation assays measure synapse assembly that is induced in cocultured neurons by a candidate synaptogenic surface protein that is expressed in a nonneuronal cell (19–21). To assess whether *Nrxn1*, *Nrxn2*, and *Nrxn3* exhibit similar synaptogenic activities in this assay, we expressed Nrxn1β, Nrxn2β, or Nrxn3β containing or lacking an insert in SS4 in human embryonic kidney 293 (HEK293) cells. After coculturing the HEK293 cells with hippocampal neurons, we quantified postsynaptic specializations formed on the HEK293 cells by staining for PSD95 (Fig. 1*A*). We analyzed both SS4 splice variants to avoid overlooking a potential effect of alternative splicing that regulates neurexins (3). All the three β-neurexins potently induced postsynaptic specializations in cocultured neurons independent of alternative splicing at SS4, with Nrxn1β and Nrxn2β being more effective than Nrxn3β (Fig. 1*B*). Thus, Nrxn2β is synaptogenic similar to Nrxn1β and Nrxn3β in the heterologous synapse formation assay.

**Fig. 1.** *Nrxn2β* potently induces heterologous synapse formation similar to *Nrxn1β* and *Nrxn3β* independent of alternative splicing at SS4. (*A*) Representative confocal images of heterologous synapse formation assays. HEK293 cells that coexpress GFP (green) and the indicated neurexin are cocultured with hippocampal neurons at DIV16. After 24 h, the cocultures are analyzed for induction of postsynaptic specializations on the HEK293 cells by immunocytochemistry for the postsynaptic marker PSD95 (red). HEK293 cells coexpress GFP (green) with no other protein (mock) or with Nrxn1β, Nrxn2β, or Nrxn3β lacking or containing an insert in SS4. (*B*) Summary graph of the synaptic PSD95 signal surrounding GFP-positive HEK293 cells as a measure of synapse formation (dashed lines = PSD95 signal in controls). Data are means ± SEMs (numbers in bars show number of cells/experiments analyzed); statistical significance was assessed by two-way ANOVA and post-hoc Tukey’s test (significance of the comparison to the control is indicated (*P < 0.05; **P < 0.01, and ***P < 0.001).

### *Nrxn2* Suppresses Excitatory Synapse Assembly in Cultured Neurons.

To analyze the physiological requirements for *Nrxn2* in cultured neurons, we infected hippocampal cultures from *Nrxn2* conditional knockout (cKO) mice with lentiviruses expressing EGFP-tagged wild-type (Cre) or mutant Cre-recombinase (ΔCre; as a control). In this manner, we studied neurons that contain precisely matching genetic backgrounds and either express or lack *Nrxn2* (22). Morphological analyses of control and *Nrxn2*-deficient neurons demonstrated that the *Nrxn2* deletion caused a robust increase (~30%) in the density of excitatory synapses as measured by immunocytochemistry with antibodies to vGluT1 and Homer1, but did not produce major effects on the intensity of these puncta (Fig. 2 *A*–*D*). This finding was independently replicated by a separate experimenter (*SI Appendix*, Fig. S1 *A* and *B*). No effect of the *Nrxn2* deletion on inhibitory synapse densities, as measured by immunocytochemistry with antibodies to vGAT, was detected (*SI Appendix*, Fig. S1 *C* and *D*). These observations are consistent with previous findings in vivo suggesting that *Nrxn2* normally inhibits, instead of promoting, excitatory synapse assembly (17). Moreover, these data indicate that the synaptogenic activity of *Nrxn2* in the heterologous synapse formation assay (Fig. 1) is misleading, thereby contradicting current ideas of neurexins as general synaptic organizers that promote synapse assembly.

**Fig. 2.** Deletion of *Nrxn2* increases excitatory synapse numbers and elevates the frequency of mEPSCs in cultured hippocampal neurons. (*A*) Representative images of cultured hippocampal *Nrxn2* cKO neurons stained for vGluT1 (excitatory presynaptic marker; red), Homer1 (excitatory postsynaptic marker; green), MAP2 (dendritic marker; magenta), and Cre/dCre-GFP (blue). (*B* and *C*) Summary graphs of the synaptic puncta density (left graphs) and synaptic puncta staining intensity (right graphs) as measured for vGluT1^+^ (*B*) and Homer1^+^ puncta (*C*). (*D*) Summary graph of colocalized vGluT1^+^ and Homer1^+^ puncta. (*E*) Representative traces of miniature excitatory postsynaptic currents (mEPSC) recorded in the presence of 1 μM tetrodotoxin. (*F*) Cumulative probability plots of mEPSC interevent intervals (*Inset*: summary graph of the mEPSC frequency) and of mEPSC amplitudes (*Inset*: summary graph of the mEPSC amplitude) showing that deletion of *Nrxn2* increases the frequency of excitatory spontaneous synaptic events. (*G*) Representative traces of miniature inhibitory postsynaptic currents (mIPSCs). (*H*) Cumulative probability plots of mIPSC interevent intervals (*Inset*: summary graph of the mIPSC frequency) and of mIPSC amplitudes (*Inset*: summary graph of the mIPSC amplitude) showing that deletion of *Nrxn2* has no effect on the frequency of inhibitory spontaneous synaptic events. Data are means ± SEMs. Sample sizes are listed in the graphs as the number of cells/experiments. Statistical assessments were performed by the Mann–Whitney test comparing ΔCre and Cre conditions (*B*–*D* and *F*–*H*), with **P < 0.01 (nonspecific comparisons are not indicated). For an independent validation of these results, see *SI Appendix*, Fig. S1.

We next tested whether the new synapses induced by the *Nrxn2* deletion in cultured hippocampal neurons were functional by performing whole-cell patch-clamp recordings. Consistent with the selective increase in excitatory synapse density, the *Nrxn2* deletion elevated the frequency but not the amplitude of spontaneous miniature excitatory postsynaptic currents (mEPSCs; Fig. 2 *E* and *F*). The *Nrxn2* deletion had no effect on miniature inhibitory postsynaptic currents (mIPSCs; Fig. 2 *G* and *H*). Again, this result was independently replicated by a second experimenter (*SI Appendix*, Fig. S1 *E*–*H*).

The mEPSC frequency depends primarily (but not exclusively) on the number and release probability of synapses of a neuron. To determine whether the *Nrxn2* deletion causes a change in synapse properties in addition to synapse numbers, we monitored evoked synaptic transmission. The *Nrxn2* deletion increased the amplitude of evoked AMPAR-EPSCs (~100%; Fig. 3 *A* and *B*) and decreased the coefficient of variation of AMPAR-EPSC amplitudes in cultured neurons (Fig. 3*C*), but did not affect the AMPAR-EPSC kinetics (Fig. 3*D*). Similarly, the *Nrxn2* deletion enhanced the amplitude of NMDAR-EPSCs (~25%; Fig. 3 *E* and *F*) and suppressed the coefficient of variation of the NMDAR-EPSC amplitude (Fig. 3*G*), again without affecting the NMDAR-EPSC kinetics (Fig. 3*H*). These observations were also independently replicated by multiple experimenters, although the relative effect sizes varied between experiments and experimenters (*SI Appendix*, Fig. S2 *A*–*C*). Consistent with no change in inhibitory synapse numbers (*SI Appendix*, Fig. S1 *C* and *D*) and mIPSCs (*SI Appendix*, Fig. S1 *G* and *H*), no effect of the *Nrxn2* deletion on evoked IPSCs was detected (*SI Appendix*, Fig. S2*D*).

**Fig. 3.** Deletion of *Nrxn2* increases the strength and presynaptic release probability of excitatory synapses in cultured hippocampal neurons, measured via the amplitude, coefficient of variation, and paired-pulse ratio of evoked EPSCs, and enhances the Ca^2+^-sensitivity of neurotransmitter release. (*A* and *B*) The *Nrxn2* deletion increases the amplitude of evoked excitatory postsynaptic currents (EPSCs) mediated by AMPARs [representative traces (*A*) and summary graph (*B*) of AMPAR-EPSCs amplitude recordings from hippocampal neurons cultured from newborn *Nrxn2* cKO mice, infected with lentiviruses expressing active (Cre) or mutant inactive (ΔCre) Cre recombinase at DIV4, and analyzed at DIV14; recordings were performed at -70 mV holding potentials]. (*C* and *D*) The Nrxn2 deletion decreases the coefficient of variation (*C*) of AMPAR-EPSCs indicative of an increased release probability but has little effect on the AMPAR-EPSC kinetics (*D*). (*E*–*H*) The *Nrxn2* deletion also increases the amplitude of evoked EPSCs mediated by NMDARs accompanied by a decrease in the coefficient of variation (*E* and *F*, representative traces (*E*) and summary graph (*F*) of NMDAR-EPSCs amplitude recordings in hippocampal neurons performed at a +40 mV holding potentials; (*G* and *H*) summary graphs of coefficient of variation (*G*) and decay time (*H*)]. (*I*–*K*) The elevated amplitude of NMDAR-EPSCs induced by the *Nrxn2* deletion is associated with a decrease in paired-pulse ratio, suggesting an increase in release probability consistent with the decrease in the coefficient of variation [*I*, representative traces of NMDAR-EPSCs evoked by two closely spaced stimuli; *J* and *K* absolute amplitudes of the first and second EPSCs (*J*) and paired-pulse ratio (*K*) as a function of the interstimulus interval]. (*L*–*O*) The *Nrxn2* deletion increases the Ca^2+^-responsiveness of excitatory synapses [*L*, representative traces of NMDAR-mediated EPSCs recorded in the presence of the indicated extracellular Ca^2+^-concentrations ([Ca^2+^]_ex_); *M*, cumulative plot of [Ca^2+^]_ex_ dependence. Summary graphs of apparent EC_50_ of [Ca^2+^]_ex_ (*N*), and Hill coefficient (*O*)]. Data are means ± SEMs. Sample sizes are listed in the graphs (cells/independent experiments). Statistical assessments were performed by the Mann–Whitney test comparing Cre to ΔCre conditions (*B*–*D*, *F*–*H*, *N*, and *O*) or by two-way ANOVA followed by post hoc Tukey's test (*J* and *K*), or Kolmogorov–Smirnov (KS) test (*M*) with *P < 0.05; **P < 0.01. For an independent validation of a subset of these results, see *SI Appendix*, Fig. S2.

The decreased coefficient of variation in *Nrxn2*-deficient neurons suggests an increase in release probability. To test this hypothesis, we measured the paired-pulse ratio of NMDAR-EPSCs (Fig. 3*I*). In these measurements, we replicated the large increase in the amplitude of NMDAR-EPSCs that persisted in the responses induced by a second, closely spaced stimulus (Fig. 3*J*) and was associated with a robust decrease in paired-pulse ratio, consistent with an increase in release probability (Fig. 3*K* and *SI Appendix*, Fig. S2*E*). To further explore the mechanistic basis for the increased release probability, we monitored NMDAR-EPSC amplitudes as a function of the extracellular Ca^2+^-concentration (Fig. 3*L*). The *Nrxn2* deletion caused a small but significant shift in the Ca^2+^-dependence of NMDAR-EPSC amplitudes (Fig. 3*M*). As a result, the apparent Ca^2+^-sensitivity of NMDAR-EPSCs was increased, as reflected in a ~20% decrease in the apparent EC_50_ for Ca^2+^ (Fig. 3*N*), whereas the apparent Ca^2+^-cooperativity was not changed (Fig. 3*O*). Thus, the *Nrxn2* deletion has two functional effects on cultured neurons: It causes an increase in the synapse density and additionally an increase in release probability that is due, at least in part, to an enhanced Ca^2+^-sensitivity of release.

### An mGluR2 Agonist Reverses the Increase in Synaptic Strength Induced by the *Nrxn2* KO.

The dual action of the *Nrxn2* deletion that we observed here, an increase in synapse numbers and in release probability, agrees well with previous in vivo data (17). It raises an important question: Does the *Nrxn2* deletion act via a single mechanism that controls both synapse numbers and the release machinery, for example by restricting the assembly of active zones that may spawn formation of new synapses, or does the *Nrxn2* deletion act by separate mechanisms that control synapse numbers and the presynaptic release probability?

As a first step to addressing this question and probing the nature of the increase in the presynaptic release probability in *Nrxn2*-deficient synapses, we measured the relative effects of an mGluR2 agonist, LY379268 (23–25), on synaptic strength (Fig. 4). As before, we examined hippocampal neurons cultured from *Nrxn2* cKO mice that were infected with lentiviruses expressing mutant Cre (ΔCre, control) and active Cre (*Nrxn2* deletion), and monitored spontaneous mEPSCs (Fig. 4 *A*–*C*) and evoked NMDAR-EPSCs using the paired-pulse stimulation paradigm to also assess the release probability (Fig. 4 *D*–*F*).

**Fig. 4.** The mGluR2 agonist LY379268 reverses the enhancement of synaptic transmission induced by the *Nrxn2* deletion in cultured hippocampal neurons. (*A*–*C*) mGluR2 stimulation reverses the increase in mEPSC frequency induced by the deletion of *Nrxn2* without significantly affecting the mEPSC amplitude (*A*, representative mEPSC traces; *B* and *C*, summary graphs of the mEPSC frequency and amplitude). (*D*–*F*) mGluR2 agonism also reverses the increase in the NMDAR-EPSC amplitude and the decrease in paired-pulse ratios induced by deletion of *Nrxn2* (*D*, representative traces; *E*, summary graph of NMDAR-EPSCs amplitude; *F*, summary graph of paired-pulse ratios). Data are means ± SEMs. Sample sizes are listed in the graphs (cells/independent experiments). Statistical assessments were performed by two-way ANOVA followed by post hoc Tukey's test, with *P < 0.05; **P < 0.01, and ***P < 0.001.

Addition of LY379268 to control neurons induced only a small decrease in mEPSC frequency that was statistically significant when assessed with a Student’s *t* test but not significant when assessed by two-way ANOVA, consistent with a relative sparsity of mGluR2’s on hippocampal synapses (Fig. 4 *A* and *B*). No effect of LY379268 on the mEPSC amplitude was detected, as would be predicted from the mode of action of mGluR2. When added to *Nrxn2*-deficient neurons, however, LY379268 reversed the dramatic increase (~150%) in mEPSC frequency, again without affecting the mEPSC amplitude (Fig. 4 *A*–*C*). Similarly, LY379268 had little effect on the amplitude and paired-pulse ratio of evoked NMDAR-EPSCs in control neurons (Fig. 4 *D*–*F*). However, LY379268 suppressed the large increase (~120%) in the amplitude of evoked NMDAR-EPSCs in *Nrxn2*-deficient neurons and reversed the decrease in paired-pulse ratio in these neurons (Fig. 4 *D*–*F*). These data confirm that the *Nrxn2* deletion produced a large increase in release probability in cultured hippocampal neurons and demonstrate that this increase is associated with a heightened sensitivity to mGluR2 activation consistent with an increased Ca^2+^-responsiveness of release. These results thus support the notion that the *Nrxn2* deletion causes a reorganization of the presynaptic release machinery toward higher efficacy, which starkly contrasts with what we observed with the neurexin-1/2/3 triple deletion (26, 27).

### *Nrxn2β* Splice Variants Differentially Rescue the Increase in Synapse Numbers and Release Probability in *Nrxn2*-Deficient Hippocampal Neurons.

We next approached the dissection of *Nrxn2* function with rescue experiments. Neurexins are extensively alternatively spliced (5, 10–12), and at least alternative splicing at SS4 that is present both in α- and β-neurexins is functionally important (13–16, 28, 29). Thus, we tested in rescue experiments Nrxn2β and not Nrxn2α constructs because Nrxn2β is smaller than Nrxn2α and has fewer splice variants (4 vs. >100; Fig. 5*A*) but binds to most of the known ligands of Nrxn2α since it also contains SS4. Moreover, Nrxn2β—like Nrxn2α—includes SS5 that contains a very large insert sequence potentially capable of multiple protein interactions (6).

**Fig. 5.** The two Nrxn2β splice variants that contain an insert in SS4 with or without an insert in SS5 revert the increased synapse density induced by the *Nrxn2* deletion, whereas the two corresponding Nrxn2β variants lacking an insert in SS4 are inactive. (*A*) Schematic of the domain structure of Nrxn2β splice variants used in rescue experiments (SP, signal peptide; TMR, transmembrane region). (*B*–*E*) Nrxn2β splice variants containing an insert in SS4 (Nrxn2β^SS4+SS5−^ and Nrxn2β^SS4+SS5+^) normalize the increased synapse numbers induced by the *Nrxn2* deletion, whereas Nrxn2β splice variants lacking an insert in SS4 (Nrxn2β^SS4−SS5−^ and Nrxn2β^SS4−SS5+^) have no effect [*B*, representative images of cultured hippocampal Nrxn2 cKO neurons with coexpression of Cre and Nrxn2β splice variants; *C* and *D*, summary graphs of the synaptic puncta density (*Left* graphs) and synaptic puncta staining intensity (*Right* graphs) as measured for vGluT1^+^ (*C*) and Homer1^+^ puncta (*D*); *E*, summary graph of puncta containing colocalized vGluT1^+^ (red) and Homer1^+^ (green) signals]; and Cre/ΔCre-GFP (blue). Data are means ± SEMs. Sample sizes are listed in the graphs (cells/independent experiments). Statistical assessments were performed by one-way ANOVA followed by post hoc Tukey's test with *P < 0.05; **P < 0.01, and ***P < 0.001.

We infected *Nrxn2*-deficient neurons with lentiviruses expressing the four *Nrxn2β* splice variants with an N-terminal HA-tag (Fig. 5*A*). We then analyzed the “rescued” neurons in comparison to control neurons or to *Nrxn2*-deficient neurons that did not express rescue constructs (Figs. 5 and 6). Surface staining confirmed that all Nrxn2β rescue proteins were efficiently transported to the neuronal cell surface (*SI Appendix*, Fig. S3; note that all rescue experiments are likely overexpression situations). We then measured the effect of the overexpression of various Nrxn2β proteins on synapse density, using double-labeling for a presynaptic (vGluT1) and a postsynaptic marker (Homer1) to ensure precise monitoring of synapses (Fig. 5*B*). Analyses of synapse numbers using either the presynaptic (Fig. 5*C*) or postsynaptic marker signals (Fig. 5*D*) or the coincidence of pre- and postsynaptic marker signals (Fig. 5*E*) demonstrated that the two *Nrxn2β* splice variants with an insert in SS4 (Nrxn2β-SS4+SS5− and Nrxn2β-SS4+SS5+) largely reversed the increase in synapse density produced by the *Nrxn2* deletion, whereas the other two splice variants without an insert in SS4 (Nrxn2β-SS4-SS5− and Nrxn2β-SS4−SS5+) did not (Fig. 5 *C*–*E*). These data suggest that *Nrxn2* restricts synapse numbers in a manner regulated by alternative splicing at SS4 but independent of alternative splicing at SS5.

We next examined the effect of the Nrxn2β protein rescue on synaptic transmission. Measurements of mEPSCs revealed, surprisingly, that only one Nrxn2β splice variant (Nrxn2β-SS4+SS5+) robustly reversed the increase in mEPSC frequency induced by the *Nrxn2* deletion, whereas the other splice variant that also rescued the synapse density phenotype (Nrxn2β-SS4+SS5−) had no effect (Fig. 6 *A* and *B*). Again, no change in mEPSC amplitude was noted (Fig. 6*C*). Finally, we analyzed evoked NMDAR-EPSCs using the paired-pulse stimulation protocol (Fig. 6*D*). Only the Nrxn2β-SS4+SS5+ splice variant reversed the large increase in NMDAR-EPSC amplitude in *Nrxn2*-deficient synapses (Fig. 6*E*) and normalized the equally large decrease in paired-pulse ratio (Fig. 6*F*). These data show that different Nrxn2 splice variants differentially rescue the *Nrxn2* KO phenotypes. Only one variant (Nrxn2β-SS4+SS5+) reversed the increased release probability and the synapse density, while another variant (Nrxn2β-SS4+SS5−) additionally normalized the increased synapse density but not the increased release probability.

**Fig. 6.** The increase in mEPSC frequency in *Nrxn2*-deficient neurons that is dependent on the number of synapses and on their release probability is reversed by both of the two Nrxn2β splice variants containing an insert in SS4 with or without an insert in SS5, whereas the increased evoked EPSC amplitude and the decreased paired-pulse ratio of evoked EPSCs in *Nrxn2*-deficient neurons that is dependent primarily on the release probability is reversed only by the Nrxn2β splice variant containing an insert in both SS4 and SS5. (*A*–*C*) The Nrxn2β splice variant containing the insert in both SS4 and SS5 (Nrxn2β^SS4+SS5+^) fully reverses the increase in mEPSC frequency induced by the *Nrxn2* deletion, whereas the splice variant lacking an insert in both SS4 and SS5 (Nrxn2β^SS4-SS5-^) has an intermediate effect, and the other two splice variants (Nrxn2β^SS4+SS5-^ and Nrxn2β^SS4-SS5+^) are inactive [*A*, representative mEPSC traces; *B* and *C*, summary graphs of the mEPSC frequency (*B*) or amplitude (*C*)]. (*D*–*F*) Only the Nrxn2β splice variant containing an insert in both SS4 and SS5 (Nrxn2β^SS4+SS5+^) reverses the increase in NMDAR-EPSC amplitudes and the decrease in paired-pulse ratio induced by the Nrxn2 deletion, whereas all the other three Nrxn2β splice variants are inactive (*D*, representative traces; *E*, summary graph of NMDAR-EPSCs amplitude; *F*, summary graph of paired-pulse ratios). Data are means ± SEMs. Sample sizes are listed in the graphs (cells/independent experiments). Statistical assessments were performed by one-way ANOVA followed by post hoc Tukey's test with *P < 0.05; **P < 0.01, and ***P < 0.001.

## Discussion

Here, we show in cultured hippocampal neurons that, similar to *Nrxn1* and *Nrxn3*, *Nrxn2* is synaptogenic in heterologous synapse formation assays (Fig. 1). However, we find that, different from *Nrxn1* and *Nrxn3*, *Nrxn2* functions to repress instead of promoting synapse formation between neurons (Figs. 2–6). Moreover, we demonstrate that *Nrxn2* restricts two separate components of synapse organization, namely the formation/maintenance of synapses and the presynaptic neurotransmitter release probability. The loss of the first component is manifested by the robust increase in synapse density (~30%) upon deletion of *Nrxn2* (Fig. 2), while the loss of the second component is manifested by the large decreases in the coefficient of variation of AMPAR-EPSCs (~50%) and NMDAR-EPSCs (~50%) and the paired-pulse ratio (~30% at 50 ms interval) upon deletion of *Nrxn2* (Figs. 2 and 3), with the increases in mEPSC frequency (~120%), AMPAR-EPSC amplitudes (~120%), and NMDAR-EPSC amplitudes (~30%), resulting from a loss of both components. Furthermore, we show that rescue with the Nrxn2β-SS4+SS5+ and Nrxn2β-SS4+SS5− splice variants of *Nrxn2* reversed the increase in synapse density in *Nrxn2*-deficient neurons (Fig. 5). In contrast, rescue with only the Nrxn2β-SS4+SS5+ but not the Nrxn2β-SS4+SS5− splice variant of *Nrxn2* normalized the increased release probability in *Nrxn2*-deficient neurons (Fig. 6). These data validate and extend our previous in vivo study identifying a role for *Nrxn2* in restricting synapse assembly (17), suggesting that the two processes restrained by *Nrxn2* in synapse assembly—synapse formation/maintenance and the presynaptic release probability—are mediated by distinct molecular pathways. Moreover, these results confirm earlier suggestions (3) that the heterologous synapse formation assay is not predictive of a physiological function in establishing synaptic connections, although this assay is useful as an approach to probe synapse organizing mechanisms (20, 30).

The overall view that emerges from these data is that neurexins are functionally more heterogeneous and complex than previously envisioned. At this point, scores of studies document diverse functions of various neurexins in different facets of synapse organization, ranging from regulating the number of synapses to determining their pre- or postsynaptic properties. However, the findings on *Nrxn2* that we report here and described earlier (17) are unexpected in revealing a major enhancement of synapse numbers by a genetic neurexin manipulation. In α-neurexin triple KO mice, a modest decrease in inhibitory but not excitatory synapse numbers was observed (30, 31), whereas in α/β-neurexin triple KO mice, most synapse numbers were unchanged although a subset of synapses exhibited decreased numbers (26, 32). In cultured neurons with α- and β-neurexin triple deletions, no gain or loss of synapses was detected (9, 33). In human neurons, *NRXN1* mutations have no effect on synapse numbers although they robustly impair synaptic transmission (34, 35). In contrast, in *Nrxn1* mutant mice lacking the heparan sulfate modification, a discrete synapse loss in the CA3 region of the hippocampus was found (36), although single deletions of *Nrxn1* have not yet been studied in mice in detail. In none of these studies—nor in the many RNAi experiments that are not easily evaluated because of their potential for artifacts—was an increase in synapse density observed.

Our current study is at odds with two previous findings. First, an earlier paper on *Nrxn2*-mutant mice suggested that the analyzed *Nrxn2* mutation caused a decrease in mEPSC frequency, no change in synapse numbers, and a decrease in paired-pulse ratios, which is puzzling phenotype since this phenotype suggests at the same time an increase and a decrease in release probability. The mice used by Born et al. (18) were generated in our laboratory but we could not determine whether the *Nrxn2* gene in these mice contained a deletion or a chromosomal gene rearrangement. It is thus possible that these mice express mutant *Nrxn2* proteins that retain some *Nrxn2* functions and may explain the phenotype observed by Born et al. (18). Such an explanation would be consistent with our observation that the two synapse-restricting *Nrxn2* deletion phenotypes, the increase in synapse numbers and in release probability, are differentially rescued by *Nrxn2* splice variants, suggesting a complex mode of action (Figs. 5 and 6). Second, a recent study proposed that *Nrxn2* regulates axonal pathfinding as a receptor for *Cbln1* (37). However, this conclusion was puzzling given that *Nrxn2*α KO mice exhibit no apparent change in axonal pathfinding (30, 31, 38), nor did we observe changes in axonal pathfinding in constitutive *Nrxn2* KO mice (17). Moreover, no axonal pathfinding defects were detected in *Cbln1* KO mice (39–42), suggesting that the observed changes in axonal pathfinding by Han et al. (37) may be specific to a particular experimental condition and not generally applicable.

However, our study also has several limitations and raises new questions. Most importantly, we are unable to explain how *Nrxn2* might restrict the formation and organization of synapses in an alternative splicing-dependent manner. The splice site-dependent reversal of the *Nrxn2* KO phenotype suggests that the binding of the *Nrxn2* ligand that mediates synapse restriction is regulated by alternative splicing. However, which of the multiple splice site-dependent ligands of neurexins might be involved and why only *Nrxn2* but not *Nrxn1* and *Nrxn3* (that also interact with the same ligands) restricts synaptic connectivity remains unclear.

Moreover, our experiments—and other studies examining synapse density—do not distinguish between synapse assembly and synapse maintenance. We do not know whether the *Nrxn2* deletion increases synapse numbers because it enhances synapse assembly or because it decreases synapse elimination. The distinction between synapse assembly and maintenance may be somewhat semantic since at least in the hippocampus, synapses turn over rapidly (43, 44). Overall synapse formation may proceed by a promiscuous assembly process that then leads to the stabilization of only those synapses that are validated. In other words, synapse assembly and maintenance may be two facets of the same process, and *Nrxn2* might act by enabling synapse elimination instead of restraining synapse formation.

As yet another limitation, our experiments only examine synapses from one brain region (the hippocampal formation) and also do not identify which synapses in this brain region are affected in our experiments. Even in cultured neurons, synapses are heterogeneous but likely retain region-specific features that may depend on the various neurexin splicing patterns in the neurons involved. It is thus possible that *Nrxn2* restricts only subsets of synapses, and that in other brain regions where other *Nrxn2* splice variants are expressed, *Nrxn2* may have other functions. Moreover, we did not compare the roles of Nrxn2α vs. Nrxn2β isoforms that are highly differentially expressed as various splice variants (10). In addition, Nrxn2α messenger ribonucleic acids (mRNAs) include a long conserved 5′ untranslated region with multiple upstream ATGs and a G-quadruplex sequence that combine to inhibit translation, suggesting additional regulation of Nrxn2α expression at the translational level (45). Furthermore, it is possible that Nrxn2α may be functionally different from Nrxn2β we examined here, another question that future experiments will have to address. As an additional question, we do not know why the *Nrxn2* deletion causes an increase in hippocampal synapse density whereas the triple Nrxn123 deletion does not (32, 33). The most parsimonious hypothesis addressing this question is that *Nrxn2* functionally interacts with *Nrxn1* and/or *Nrxn3*. However, other explanations are possible, such as a differential regulation of a common downstream target. As a finding, the role of *Nrxn2* in restricting synaptic connections thus raises a panoply of questions that will need to be addressed in future experiments.

In summary, our data are consistent with the concept of neurexins as master regulators of synapse organization, but our data also suggest that their action is not what one would expect of a homologous family of proteins with similar functions. Instead, our data support the emerging notion that different neurexins perform diversified roles that are regulated by alternative splicing and critically contribute to the functional architecture of synapses. It is astounding to perceive how many profound regulatory actions are performed by neurexins. Thus, homologous genes can mediate multifarious functions depending on the cellular context of their expression, their alternative splicing, and the presence of various ligands. Deconstructing the physiological activities and mechanisms of neurexins will be a continuing challenge for future experiments, but likely rewarding as their functions appear to be at the center of what constitutes a synapse and shapes its properties.

## Methods

### *Nrxn2* cKO Mice and Mouse Husbandry.

*Nrxn2* (cKO) mice were described previously (17). In brief, these mice contain loxP-sites flanking exon 18, the first common exon of *Nrxn2α* and *Nrxn2β* whose deletion abolishes the reading frame of all *Nrxn2* transcripts. Deletion of exon 18 results in the production of truncate unstable *Nrxn2* protein and in the degradation of the *Nrxn2* mRNA by nonsense-mediated decay. All mouse procedures were approved by animal use committees at Stanford University.

### Heterologous Synapse Formation Assays.

Heterologous synapse formation assays were performed essentially as described (21, 46, 47). Hippocampal neurons cultured from neonatal wild-type mice were cocultured at DIV16 with the transfected HEK293 cells expressing EGFP without or with coexpression of various β-neurexins. After 24 h, cells were fixed with 4% paraformaldehyde (PFA) and immunostained with mouse anti-PSD95 (SySy; 1:500). Species-specific AlexaFluor-546 conjugated antibodies (Invitrogen; 1:500) were used as secondary antibodies.

### Neuronal Cultures.

Neuronal cultures were obtained from mouse hippocampus as described (13). In brief, mouse hippocampi were dissected from newborn mice and dissociated in medium containing papain (10 U/mL) for 20 min at 37 °C. Cell suspensions were filtered, plated on matrigel-coated circular glass coverslips (diameter = 12 mm), and cultured in Neurobasal-A (GIBCO) supplemented with B27 (GIBCO), L-glutamine, and 2 µM Ara-C (Sigma). Neurons were infected at DIV4 with lentiviruses expressing EGFP-tagged Cre (test) or ΔCre (mutant control) (22) that contain a nuclear localization signal and HA-tagged *Nrxn2β *splice variants (Nrxn2β-SS4−SS5−, Nrxn2β-SS4−SS5+, Nrxn2β-SS4+SS5−, and Nrxn2β-SS4+SS5+) as described previously (13), but were modified with the addition of an N-terminal HA-tag following the signal peptide. All lentiviral expressions were driven by the human synapsin-1 promoter. We assessed the infection efficacy of neurons (>90%) via their nuclear EGPF fluorescence and confirmed that Cre recombinase excised the corresponding exon(s) in the hippocampal cultured neurons using genomic PCR. HA-surface staining was used to validate the surface expression of Nrxn2β splice variants (*SI Appendix*, Fig. S3).

### Viral Production.

Lentivirus constructs and virus preparation from HEK cells were done as previously described (13). HEK-293T cells were cotransfected with three packaging plasmids (pCMV-VSVG, pMDLg/pRE, and pRSV-REV) using the calcium phosphate method (13, 22). Supernatants containing the lentiviruses were harvested 48 to 72 h after transfection and added to cultured neurons.

### Immunocytochemistry.

Neuronal cultures were prepared for immunofluorescence essentially as described (13, 32). Cultures were fixed with 4% PFA at DIV14. Neuronal cultures on glass coverslip were washed with PBS and permeabilized in 0.3% Triton X-100/PBS for 5 min at RT. Unpermeabilized samples were used in surface staining. Cells were subsequently incubated in blocking solution (5% goat serum in PBS) for 1 h at RT under gentle agitation and incubated for 12 h at 4 °C with primary antibodies diluted in blocking solution (anti-vGluT1, 1:1,000, guinea pig, Millipore; anti-vGAT, 1:500, rabbit, Millipore; anti-MAP2, 1:1,000, mouse, Sigma or chicken, EnCor; anti-PSD95, 1:1,000, mouse, Thermo Fisher Scientific; anti-Homer, 1:1,000, rabbit, Millipore; anti-HA, 1:1,000, rabbit, Millipore). Neuronal cultures were washed in PBS, treated with species-specific secondary antibodies (1:1,000, Alexa 488, 545, 633, Invitrogen) at RT for 1 h, and washed again in PBS. The glass coverslips were then mounted on superfrost slides and covered with mounting media (Vectashield, Vector Labs). The infected neurons were randomly chosen and acquired using a Nikon confocal microscope (A1Rsi). Acquisition and quantitative analyses were carried out on an average of 10 to 12 neurons per condition per animal. Single-plane confocal images (1,024 × 1,024 resolution) were acquired with a 60× oil objective (PlanApo, NA1.4). All acquisition parameters were kept constant among different conditions within experiments. Image backgrounds were normalized, and immunoreactive elements were analyzed with Nikon analysis software automatically without operator input.

### Culture Electrophysiology.

Hippocampal cultured neurons were recorded at DIV 14-17 (13). Electrophysiology recordings were performed at room temperature, performed in whole-cell patch-clamp mode using concentric extracellular stimulation electrodes. The glass pipettes (2 to 3 MΩ filled with intracellular pipette solution) were pulled from borosilicate glass capillaries with a vertical micropipette puller (PC-10, Narishige). After formation of the whole-cell configuration and equilibration of the intracellular pipette solution, the series resistance was adjusted to 8 to 12 MΩ. Synaptic currents were monitored with a Multiclamp 700B amplifier (Molecular Devices). A bipolar stimulation electrode (FHC, Bowdoinham, ME) was placed 100 to 150 µm from the soma of the neurons recorded to apply focal square pulse stimuli (duration 1 ms) and trigger evoked synaptic responses. The frequency, duration, and magnitude of the extracellular stimulus were controlled with a Model 2100 Isolated Pulse Stimulator (A-M Systems) synchronized with Clampex 9 data acquisition software (Molecular Devices). The whole-cell pipette solution contained (in mM): 120 CsCl, 5 NaCl, 1 MgCl_2_, 10 HEPES, 10 EGTA, 0.3 Na-GTP, 3 Mg-ATP, and 5 QX-314 (pH 7.2, adjusted with CsOH). The bath solution contained (in mM): 140 NaCl, 5 KCl, 2 MgCl_2_, 2 CaCl_2_, 10 HEPES, and 10 glucose (pH 7.4, adjusted with NaOH). Spontaneous mIPSCs and mEPSCs were monitored in the presence of tetrodotoxin (TTX, 1 μM). Miniature events were analyzed in Clampfit 9 (Molecular Devices) using the template-matching search and a minimal threshold of 5 pA, and each event was visually inspected for inclusion or rejection by an experimenter blind to the recording condition. IPSCs, as well as AMPA- or NMDA-receptor-mediated EPSCs, were pharmacologically isolated by adding blockers against AMPA receptor (CNQX, 10 μM), NMDA receptor (AP-5, 50 μM), or GABA_A_ receptor (picrotoxin, 50 μM) to the extracellular solution. Two pulses at different intervals (50, 100, 300, 1,000 ms and 6 s) were delivered to calculate paired-pulse ratios (PPRs). LY379268 (1 μM), mGluR2 agonist, was applied for 5 min to the neuronal culture before mEPSC or PPR measurements. All drugs were obtained from Tocris (Minneapolis, MN, USA).

### Statistical Analyses.

Intergroup comparisons were done by unpaired Mann–Whitney test. For multiple comparisons, data were analyzed with one-way or two-way ANOVA with Tukey's post-test; for cumulative distributions, Kolmogorov–Smirnov tests were used. The levels of significance were set as *P < 0.05; **P < 0.01; ***P < 0.001. Data were represented as means ± SEM.

## Supplementary Material

Appendix 01 (PDF)

Dataset S01 (XLSX)

## Data Availability

All study data are included in the article and/or *SI Appendix*.
